The article "Screening and Biological Function Analysis of miRNA and mRNA Related to Lung Adenocarcinoma Based on Bioinformatics Technology" was published in 2022. Journal: J Oncol.

# Screening and Biological Function Analysis of miRNA and mRNA Related to Lung Adenocarcinoma Based on Bioinformatics Technology

**DOI:** 10.1155/2022/4339391

**Published:** 2022-08-31

**Authors:** Kaining Jia, Xiaocang Ren, Yuee Liu, Jiawei Wang

**Affiliations:** ^1^Clinical Trials Center, Huabei Petroleum Administration Bureau General Hospital, Renqiu 062550, China; ^2^Oncology Department, Huabei Petroleum Administration Bureau General Hospital, Renqiu 062550, China; ^3^Department of Imaging Medicine, Huabei Petroleum Administration Bureau General Hospital, Renqiu 062550, China

## Abstract

**Objective:**

To screen the differentially expressed miRNAs (DEMs) and the differentially expressed gene mRNAs (DEGs) in lung adenocarcinoma (LUAD) from the TCGA database and to explore the relationship between miRNAs and the prognosis of lung adenocarcinoma and their biological functions.

**Methods:**

The RNA-seq and miRNA-seq data of lung adenocarcinoma samples were downloaded from the TCGA database for analysis, and the R program was used to screen for differentially expressed miRNAs and mRNAs. Then, the molecular functions, biological processes, cellular components, and signaling pathways involved in the occurrence and development of LUAD were analyzed using the functional accumulation analysis software of GSEA. The relationship between the integrated differentially expressed RNAs was analyzed by miRcode, TargetScan, and miRTarbase databases, and the miRNA-mRNA network was constructed.

**Result:**

A total of 516 differentially expressed miRNAs and 5464 differentially expressed mRNAs were identified in LUAD. The GSEA enrichment analysis showed that miRNAs and mRNAs were mainly enriched in extracellular structure organization, external encapsulating structure organization, extracellular matrix organization, and gated channel activity. They were mainly involved in neuroactive ligand-receptor interaction signaling pathway. Some miRNAs and mRNAs in clustering modules were found to be associated with the prognosis of LUAD. Four targeting networks consisting of 22 miRNAs and 531 mRNAs were constructed.

**Conclusion:**

The miRNA and mRNA related to the prognosis of LUAD were screened out, which provided a valuable preliminary basis for the follow-upin-depth clinical research and basic experimental research of LUAD.

## 1. Introduction

LUAD is one of the most common malignancies with high morbidity and mortality worldwide [1]. Lung cancer is histologically divided into SCLC and NSCLC, the latter accounting for approximately 85% of total cases [2]. LUAD and LUSC are the two most common subtypes of NSCLC. The most common predominant histological subtype of LUAD is papillary (37%), followed by alveolar (30%), solid (25%), and fine bronchoalveolar (7%) carcinomas, but not pure [3]. The lung's adenocarcinoma can be classified according to the malignancy of the disease and the extent of the lesion as preinfiltrative, microinfiltrative, and invasive adenocarcinoma, with preinfiltrative lesions classified as atypical adenomatous hyperplasia and adenocarcinoma in situ [4]. The lungs are the most important sites of gas exchange in the body, and the alveoli are densely packed with capillaries that expel carbon dioxide and take in oxygen [5]. Tissue cells in the lungs may undergo DNA damage if they are exposed to carcinogens inhaled with the air, and although human tissues have the ability to repair themselves, the risk of cellular carcinogenesis increases significantly if the DNA damage is long-term and repeated [6]. Lung adenocarcinoma is the uncontrolled malignant proliferation of genetically mutated cancer cells in the lung, which invade adjacent normal tissues and form cancerous lesions [7]. Moreover, the rich vascularity of the lung facilitates the dissemination of cancer cells to the whole body through blood circulation. Hence, patients with advanced lung cancer are often accompanied by multiorgan metastases [8]. To date, the most important known lung carcinogenic factor is cigarette smoke, including active smoking or secondhand smoke exposure [9]. Risk factors that are clinically relevant to the development of lung adenocarcinoma are as follows: female, middle-aged and elderly population over 40 years of age, long-term heavy smoking, long-term exposure to heavy air pollution, family history, risk of occupational exposure, and concomitant chronic respiratory disease [10].

The oncogenic process of LUAD is a multistage and multigene process, involving the activation of oncogenes and inactivation of oncogenes [11]. Its treatment has changed considerably in recent years as a result of a better understanding of the biological mechanisms and the implementation of molecular and clinical biomarkers to guide clinical decisions. Despite advances in the treatment of LUAD, including surgical resection, chemotherapy, and immunotherapy, the prognosis of advanced LUAD remains poor, especially in patients with metastatic diseases [12]. The clinical presentation of the tumor is closely related to its stage and grading. The tumor, lymph node, and metastasis (TNM) staging system provides a method for assessing cancer status and predicting prognosis, and it is widely used in clinical practice [13]. Therefore, exploring the target molecules associated with TNM staging is important for the diagnosis and treatment of LUAD [14, 15].

GO is a database created by the Gene Ontology Consortium to establish a semantic vocabulary standard for qualifying and describing gene and protein functions that is applicable to a wide range of species [16] and can be updated as research progresses [17]. KEGG is a functional enrichment, i.e., a set of genes (multiple genes) that may be significantly concentrated in which functions, or arguably, in which pathways. Similar pathway databases are wikipathway, reactome, etc. The large public transcriptome database provides a valuable resource for the analysis of genome-wide coexpression networks, the screening of tumor markers associated with prognosis and phenotype, and the study of the molecular mechanisms of pathogenesis [18]. *R* package for weighted correlation network analysis (WGCNA) is a systems biology approach for describing correlation patterns between genes by microarray samples [19].

Currently available LUAD markers do not have sufficient predictive power. Most of the current methods are invasive. Therefore, we reanalyzed the TCGA dataset to find new biomarkers that are closely related to the patient TMN stage, survival rate, and other prognosis.

In this study, we downloaded raw expression data from LUAD RNA high-throughput sequencing (RNA-HTSeq) from TCGA and analyzed DEGs and DEMs between LUAD patients and normal lung gland tissues. The WGCNA approach based on DEG identified important gene coexpression modules and genes associated with TNM staging. GO and KEGG enrichment analyses were performed to analyze the functional genes and cellular signaling pathways involved. In addition, modular gene networks were constructed, and hub genes associated with TNM staging were identified by Cytoscape software. The relationship between hub genes and survival was analyzed. Four target networks consisting of 22 miRNAs and 531 mRNAs were constructed, which may be related to the development and clinical features of LUAD, laying a theoretical foundation for further research and discovery of new target biomarkers for LUAD.

## 2. Materials and Methods

### 2.1. Workflow

The workflow chart of all experimental contents in this study is shown in Figure 1. Firstly, we downloaded the dataset of LUAD experimental group and normal control group samples needed for the study from TCGA database, screened out DEMs and DEGs, and did the analysis in terms of differentially expressed miRNAs, molecular functions of mRNAs and upstream and downstream signaling pathways involved. Hub gene is often an important action target, and a research hotspot can be constructed with the coexpression of the interactions network, and then based on Hub gene is often an important target and research hotspot. Then, DEMs and DEGs are distinguished into different modules to assess whether there is a positive or negative regulatory relationship between modules and between modules and tumor malignancy degrees. The targeting network relationship between miRNAs and mRNAs was mapped.

### 2.2. Data Collection and Preprocessing

RNA-HTSeq and clinical information data of LUAD patients were downloaded from The Cancer Genome Atlas (TCGA, https://cancergenome.nih.gov/). After the removal of duplicate and no clinically informative samples, miRNA data sample profiles are as follows: 470 cancer samples and 44 normal samples, while mRNA data sample profiles are as follows: 477 cancer samples and 53 normal samples. RNA-seq data were generated by Illumina HiSeq platform. Read counts were used to indicate gene expression levels [20]. Data were processed using RStudio software (v1.1.463, Boston, USA) and in accordance with TCGA policies on human subject protection and data access.

### 2.3. Identification of DEMs and DEGs

The *R* package edgeR is used to demonstrate DEMs and DEGs between tumor and normal samples [21]. After the *p*-value is obtained, multiple hypothesis test correction is performed, and the threshold of the *p*-value is determined by controlling the FDR (false discovery rate). At the same time, we calculated the fold of differential expression according to the FPKM value, i.e., fold-change. The screening indicators for this analysis were *p*-value <0.05, log2FC > 1 or <-1.

### 2.4. GSEA Functional Enrichment Analysis

GSEA version 2.2.2 software was used for functional enrichment analysis. The miRNAs were divided into high and low expression groups according to their target molecule mRNA expression, and each expression group was enriched by the GSEA software for the Kyoto encyclopedia of genes and genomes (KEGG) signaling pathway analysis. The gene enrichment analysis was performed by default weighted enrichment statistics, and the number of random combinations was set to 1000. Gene sets with false discovery rate (FDR) < 0.25 were considered significantly enriched gene sets in GSEA.

### 2.5. WGCNA Analysis

The weighted gene coexpression network analysis is a systems biology method used to describe gene association patterns between different samples, which can be used to identify gene sets with high covariation, and it is based on the interconnectivity of gene sets and the relationship between gene sets and phenotypes. The association identifies candidate biomarker genes or therapeutic targets. WGCNA can be used to identify the cluster modules of highly correlated genes for summarizing such clusters using module signature genes (ME) or hub genes within the modules, correlating modules to each other and to external sample features (e.g., TNM staging), and using to calculate module membership metrics. WGCNA is divided into two parts: expression cluster analysis and phenotype association, which mainly include the following four steps: the calculation of correlation coefficient between genes, determination of gene modules, coexpression network, and association between modules and traits. The first step is to calculate the correlation coefficient (Person Coefficient) between any two genes. To measure whether two genes have similar expression patterns, it is generally necessary to set a threshold for screening, and those above the threshold are considered to be similar. In WGCNA analysis, the weighted value of the correlation coefficient is used, i.e., the gene correlation coefficient is taken to the power of *N*, so that the connection between the genes in the network obeys the scale-free network distribution. This algorithm has more biological significance. The second step is to construct a hierarchical clustering tree through the correlation coefficient between genes. Different branches of the clustering tree represent different gene modules, and different colors represent different modules. Based on the weighted correlation coefficients of genes, the genes are classified according to their expression patterns, and genes with similar patterns are grouped into a module. In this way, genes can be divided into dozens of modules by gene expression patterns, which is a process of extracting and summarizing information.

### 2.6. Differential Expression miRNA Gene Targeting Prediction

The so-called seed sequence (2^nd^–7^th^ nt) located at the 5′ end of the miRNA can form Watson-Crick pairing with the 3′ UTR of the target gene. It is the most important factor in the prediction of all miRNA target genes. MiRNA inhibits target gene expression at the post-transcriptional level through partial complementary pairing with the mRNA of the target gene. Studies have shown that miRNAs are involved in various biological processes, including cell proliferation, apoptosis, differentiation metabolism, development, and tumor metastasis, among other biological processes.

MiRanda it is the first miRNA target gene prediction software. Its screening of 3′ UTR is mainly based on sequence matching, thermal stability of miRNA and mRNA duplexes, and cross-species conservation of target sites. The scope of application is wide. For potential hybridization sites, miRanda also gives scores. MiRanda selects the top 10 genes in the relative 3′UTR of each miRNA as the candidate target genes for miRNAs. For multiple miRNAs corresponding to the same target site, miRanda selects the pair with the highest score and lowest free energy. The coexpression network relationship map was drawn.

## 3. Result

### 3.1. LUAD DEMs and DEGs Screened from the GEO-TCGA Database

The transcriptome data of 470 cases of miRNA cancer samples and 44 cases of normal samples were downloaded from GEO and TCGA databases, and DEMs between LUAD patients and healthy individuals were analyzed using edgeR and limma, and a total of 516 DEMs were screened, of which 203 were upregulated and 313 were downregulated (Figure 2(a)). TCGA database download of LUAD clinical mRNA data sample status is as follows: 477 cancer samples and 53 normal samples. DEGs between LUAD patients and healthy individuals were analyzed using edgeR and limma, and a total of 5464 DEGs were screened, of which 3379 were upregulated and 2085 were downregulated (Figure 2(b)).

### 3.2. GO and KEGG Enrichment Analysis

To further elucidate the biological processes, cellular components, molecular functions, and signaling pathways associated with module-trait, we applied several modules with significant module-trait relationships for GO and KEGG enrichment analysis.

The molecular functions of differentially expressed miRNA in lung adenocarcinoma were mainly enriched in channel activity, passive transmembrane transporter activity, and gated channel activity (Figure 3(a)). The cellular components were mainly enriched in the transmembrane transporter complex and collagen-containing extracellular matrix (Figure 3(a)). Biological processes were mainly enriched in extracellular structure organization, external encapsulating structure organization, and extracellular matrix organization (Figure 3(a)). The miRNA signaling pathway is mainly enriched in neuroactive ligand-receptor interaction (Figure 3(b)). The molecular functions of differentially expressed mRNA in lung adenocarcinoma were mainly enriched in channel activity, passive transmembrane transporter activity, and gated channel activity (Figure 3(c)). The cellular components were mainly enriched in collagen-containing extracellular matrix and transmembrane transporter complex (Figure 3(c)). Biological processes were mainly enriched in extracellular structure organization, external encapsulating structure organization, and extracellular matrix organization (Figure 3(c)). Lung adenocarcinoma differentially expressed mRNA signaling pathways that were mainly enriched in the neuroactive ligand-receptor interaction (Figure 3(d)). The GO and KEGG enrichment analysis of miRNAs and mRNAs differed in detail, however, the overall trends and specificities were highly consistent.

### 3.3. Construction of LUAD-Weighted Gene Correlation Network Analysis WGCNA

A biological approach to systematically characterize gene association patterns between different samples and allow the identification of highly covariant genomes. Candidate biomarker genes or therapeutic targets are identified based on the cohesion of the genome and the association between the genome and phenotype. Based on the WGCNA-based systems biology approach, gene coexpression networks were constructed to screen potential biomarkers and therapeutic targets for the disease.

In the study, a weighted gene association network was constructed using 1575 DEMs and 514 LUAD samples, and a weighted gene association network was constructed using 5464 DEMs and 530 LUAD samples. To construct the WGCNA network, we first computed the soft threshold power *β* and boosted the coexpression similarity to compute the adjacency. WGCNA adopts the pick Soft Threshold function to analyze the network topology. In the subsequent analysis, the soft threshold power *β* was set to 3, the scale independence reached 0.9, and the average connectivity was relatively high (Figure 4(a), 5(a)).

We constructed gene networks and identified modules using the one-step network construction function of the WGCNA *R* package. As shown in Figure 4, 18 coexpressed gene modules were identified by the WGCNA method, and each module was color-coded. Gray default genes cannot be classified into any modules. When there are too many genes in the grey module, previous gene screening expression matrix procedures may not be suitable (Figure 4(b)). MEgray contains genes that do not belong to any module, and it is the largest module. We analyzed the connectivity of eigengenes (eigen- + gene: a matrix of genes and samples). Intrinsic genes provide information about the relationship between the pairs of gene coexpression modules. The clustering of eigengenes indicated that these 18 modules could be divided into two groups (Figure 4(e)). In the module, MEred was significantly positively correlated with MEblack and MEmidnightblue, while MEred was negatively correlated with MEturquoise and MEgreen (Figure 4(c)). As shown in Figure 5(b), 15 coexpressed gene modules were identified by the WGCNA method, and each module was color-coded. MEturquoise is the largest module. The clustering of eigengenes indicated that these 15 modules could be divided into two groups (Figure 5(e)). Among modules, MEpurple was significantly positively correlated with MEpink and MEyellow, while MEblack was negatively correlated with MEpurple, MEblue, and MEyellow (Figure 5(c)).

Since ME can recapitulate gene expression profiles, the correlation between ME and TNM stage was calculated, called module-trait relationship analysis. To identify the module-trait relationships of gene modules, we assigned genes into corresponding modules with reference to the initially constructed modules. The correlation of each module with clinical parameters was calculated using a function of the WGCNA module eigengenes [12]. In addition, *p* ≤ 0.05 was statistically significant. As shown in Figure 4(d), MEpink was negatively correlated with the *N* phase of LUAD (*r* = −0.093, *p*=0.04). MElightcyan was positively correlated with *M* phase with LUAD (*r* = −0.093, *p*=0.04). MEsalmon was positively correlated with the total stage of LUAD (*r* = 0.12, *p*=0.007). As shown in Figure 5(d), MEbrown was negatively correlated with the *T* phase and the total Stage of LUAD (*r* = −0.11, *p*=0.02). MEred was negatively correlated with the stage with LUAD (*r* = −0.096, *p*=0.04). MEpink was positively correlated with the total stage of LUAD (*r* = 0.11, *p*=0.01). MEturquoise was positively correlated with the total stage of LUAD (*r* = 0.13, *p*=0.006).

### 3.4. A Map of the Targeting Network between LUAD miRNA and mRNA

The target mRNAs of miRNAs were searched from miRTarBase, miRDB, and TargetSsan databases to construct a targeting network consisting of differentially upregulated and downregulated miRNA-mRNAs, and the analysis was visualized using Cytoscape software.

One miRNA in M-phase targets 159 mRNAs (Figure 6(a)), of which 91 are upregulated and 68 are downregulated, and one hub miRNAs is as follows: hsa-miR-6860. Four miRNAs in N-phase target 136 mRNAs (Figure 6(b)), of which 77 are upregulated and 59 are downregulated, and four hub miRNAs are as follows: Hsa-miR-2682-3p, hsa-miR-2682-5p, hsa-miR-503-5p, and hsa-miR-503-3p. 2 miRNAs in stage phase targeted and regulated 145 mRNAs (Figure 6(c)), of which 77 were upregulated and 68 were downregulated, and the 2 hub miRNAs were as follows: hsa-miR-216b-3p and hsa-miR-216b-5p. 15 miRNAs in T-phase targeted to regulate 91 mRNAs (Figure 6(d)), of which 75 were upregulated and 16 were downregulated. 15 hub miRNAs were as follows: hsa-miR-939-5p, hsa-miR-1247-5p, hsa-miR-939- 3p, hsa-miR-6726-5p, hsa-miR-6510-5p, hsa-miR-326, hsa-miR-3615, hsa-miR-6892-3p, hsa-miR-3677-3p, hsa-miR-1247-3p, hsa-miR-99b-3p, hsa-miR -3677-5p, hsa-miR-4664-5p, hsa-miR-4736, and hsa-miR-6892-5p.

Four targeting networks consisting of 22 miRNAs and 531 mRNAs were constructed.

### 3.5. Key Gene Screening

To identify key genes, the DEGs of several modules with significant module-trait relationships were analyzed. Using Cytoscape's cytohubba plugin, key genes were screened out by the degree algorithm. Three key genes were obtained in the MEgrey60 module, which are as follows: CDCA8, KIF23, and CDT1 (Figure 7(a)). The key genes of the MElightcyan module are KIF23, CDCA8, and CCNB2 (Figure 7(b)). The key genes of the MEsalmon module include CDH1, CDH13, DAPK1, and ITGB3 (Figure 7(c)). The key genes of the MEyellow module are CDC45, KIF2C, and NCAPG (Figure 7(d)).

### 3.6. Overall Survival

The key genes of LUAD's overall survival analysis samples were divided into high expression group and low expression group. Compared with the median value of key genes, the expression survival analysis showed that ITGB3, DAPK1, CDH13, and CDH1 had no significant difference in the OS rate with patients (*p* > 0.05, Figure 8). KIF23, CDT1, CDCA8, CCNB2, NCAPG, KIF2C, and CDC45 were negatively correlated with the OS rate of patients (*p* < 0.05, Figure 8).

## 4. Discussion

With the popularity of high-resolution CT scans and the improvement of patients' health awareness, the detection rate of pulmonary nodules continues to increase. However, distinguishing benign from malignant pulmonary nodules and identifying different subtypes of NSCLC remain major challenges for clinicians. Some miRNA-mRNA regulatory changes occur at different stages of carcinogenesis. In the early diagnosis of cancer, the detection of new miRNA changes may serve as a new prognostic tumor marker method for LUAD. With advances in high-throughput sequencing technologies, the amount of transcriptome data in public databases has grown exponentially, providing ample data for screening ideal diagnostic biomarkers and evaluating their performance. In the present study, we systematically analyzed the transcriptome data of LUAD in the TCGA and GEO databases. Twenty-two miRNAs were identified and validated as possible LUAD-specific prognostic diagnostic biomarkers. Compared with previous studies, the data patient sample size in our study reached more than 1000. Therefore, our advantage lies in a wider range of candidate miRNA-mRNAs. Therefore, it is of great significance for the prognosis and treatment of LUAD to elucidate the occurrence and development mechanism of LUAD and find biomarkers that can be used for early clinical diagnosis and prognosis.

This study employed a systems biology approach, WGCNA, to identify gene modules associated with DEG and TNM staging of LUAD. A total of 1575 DEMs and module-trait relationships were identified. As shown in Figure 3(d), among the differentially expressed miRNAs, MEpink was negatively correlated with the *N*-phase of LUAD. MElightcyan is positively correlated with the *M* phase of LUAD. MEsalmon is positively correlated with the total stage of LUAD. Among the differentially expressed mRNAs, MEbrown was negatively correlated with the *T* phase of LUAD. Mered and MEbrown were negatively correlated with the stage phase of LUAD. MEpink and MEturquoise were positively correlated with the total stage of LUAD. It is suggested that these modular signature genes play an important role in the occurrence and development of LUAD.

In addition, GO and KEGG pathway enrichment analysis was performed on the module eigengenes. GO analysis showed that the differentially expressed miRNAs in lung adenocarcinoma were mainly enriched in biological processes and molecular functions. Biological process BP is mainly enriched in extracellular structural tissue, external encapsulated structural tissue, and extracellular matrix tissue. Molecular function MF is mainly enriched in channel activity, passive transmembrane transporter activity, and gated channel activity. The cellular components CC were mainly enriched in the following: transmembrane transporter complexes and extracellular matrix containing collagen. In the KEGG pathway analysis, we found that the signaling pathway was mainly enriched in neuroactive ligand-receptor interactions.

Previous studies have shown that the biological processes of lung adenocarcinoma and glioma are mainly enriched in extracellular structural tissue, external encapsulated structural tissue, and extracellular matrix tissue [22, 23]. Molecular functions in bladder cancer studies have been mainly concentrated in channel activity, passive transmembrane transporter activity, and gated channel activity [24]. Transmembrane transporter complexes and collagen-containing extracellular matrix are associated with colon cancer [25]. A neuroactive ligand-receptor interaction, a *G*protein-coupledreceptor-mediated signaling pathway, has been implicated in the progression of cancers, such as bladder and pancreatic cancer [26–28]. It regulates the axis LOC134466/hsa-miR-196a-5p/TAC1, which activates neuroactive ligand-receptor interactions by activating TACR3 in endometrial cancer (EC) [29]. In our study, it was found that the neuroactive ligand-receptor interaction signaling pathway may also have a significant relationship with the occurrence and development of lung adenocarcinoma.

After identifying the GO and KEGG enrichment analysis of LUAD-related module eigengenes, a gene network was constructed based on WGCNA to analyze the correlation between module eigengenes. Meanwhile, core miRNAs were identified using the Cytohubb package, and they are as follows: hsa-miR-6860, hsa-miR-2682-3p, hsa-miR-2682-5p, hsa-miR-503-5p, hsa-miR-503-3p, hubhsa-miR-216b-3p, hsa-miR-216b-5p, hsa-miR-939-5p, hsa-miR-1247-5p, hsa-miR-939-3p, hsa-miR-6726-5p, hsa-miR-6510-5p, hsa-miR- 326, hsa-miR-3615, hsa-miR-6892-3p, hsa-miR-3677-3p, hsa-miR-1247-3p, hsa-miR-99b-3p, hsa-miR-3677-5p, hsa-miR-4664-5p, hsa-miR-4736, and hsa-miR-6892-5p. They may be potential biomarkers to predict the prognosis of LUAD patients. In addition, potential target gene transcriptions were validated in databases, in which some target gene mRNAs were significantly downregulated/upregulated in lung adenocarcinoma tissues. These findings may provide the fundamental evidence for the future identification of potential biomarkers or anticancer targets.

Gene modules of these central genes were identified as primarily associated with the clinical metastasis of lung adenocarcinoma. Previous literature suggested that the MIR2682 locus is associated with perineural invasion in head and neck cancer [30]. MiR-2682-5p/HOXB8 promotes cell proliferation and migration in pancreatic cancer cell carcinoma [31]. The miR-2682-5p feedback loop promotes bladder cancer cell growth [32]. Ultrasonic microbubble-mediated downregulation of miR-503-5p inhibits CRC progression *in vitro* by promoting SALL1 expression [33]. Hsa_circ_0072387 inhibits the proliferation, metastasis, and glycolysis of oral squamous cell carcinoma cells by downregulating miR-503-5p [34]. LncRNADLGAP1-AS2 regulates miR-503/cyclinD1 to promote nonsmall cell lung cancer cell proliferation [35]. MiRNA-216b expression was negatively correlated with 18F-FDG uptake in NSCLC [36]. The overexpression of microRNA-939-5p contributes to cell proliferation and is associated with poor prognosis in glioma [37]. MicroRNA-939-5p directly targets IGF-1R and suppresses the aggressive phenotype of osteosarcoma by inactivating the PI3K/Akt pathway [38]. The knockdown of miR-939 may inhibit cell proliferation and invasion by regulating the expression of TIMP2 in NSCLC cells, and miR-939 may be a potential target for the treatment of NSCLC, although it requires further study [39]. MiR-1247-5p exerts a tumor suppressor effect in human astroglioma cells by targeting CDC14B [40]. Tumor-derived exosomal miR-1247-3p induces cancer-associated fibroblast activation to promote the lung metastasis of liver cancer [41]. MiR-3615 expression level in HCC patients was negatively correlated with the overall survival time, and it is positively correlated with high TNM stage, serum Ki-67 expression level, and serum alpha-fetoprotein level [42]. MiR-3677-3p promotes hepatocellular carcinoma progression by inhibiting GSK3*β* [43]. Hypoxia-induced miR-3677-3p promotes the proliferation, migration, and invasion of hepatoma cells by inhibiting SIRT5 [44]. MiR-4736 is in a region with high levels of genomic amplification in breast cancer [45]. These miRNAs may be promising novel biomarkers and prognostic factors.

It is worth mentioning that the key roles of these 22 hub miRNAs in LUAD are only predicted based on the WGCNA theory, and if verified, our findings may provide evidence for the study of anticancer targets in LUAD patients.

## 5. Conclusion

In conclusion, we identified gene modules and hub genes associated with the TNM rank using the WGCNA approach. A total of 516 differentially expressed miRNAs and 5464 differentially expressed mRNAs were identified in LUAD. GSEA enrichment analysis showed that miRNAs and mRNAs were mainly enriched in extracellular structure organization, external encapsulating structure organization, extracellular matrix organization, and gated channel activity, and it is mainly involved in the neuroactive ligand-receptor interaction signaling pathway. It was found that miRNAs and mRNAs in some clustering modules were associated with the prognosis of LUAD, and 4 targeting networks consisting of 22 miRNAs and 531 mRNAs were constructed. Mechanistically, these molecular genes may contribute to the development of changes in lung adenocarcinoma by regulating the pathways.

## Figures and Tables

**Figure 1:** Workflow.

**Figure 2:** DEMs and DEGs of cancer patients and normal groups screened in GEO and TCGA databases. All upregulated (red) and downregulated (blue) DEMs screened from GEO and TCGA databases (a), and all upregulated (red) and downregulated (blue) DEGs screened from GEO and TCGA databases (b).

**Figure 3:** DEMs and DEGs analysis of GO and KEGG. DEMs analysis of GO and KEGG, GO terms, (a) and KEGG enrichment analysis (b). DEGs analysis of GO and KEGG and GO terms, (c) and KEGG enrichment analysis (d). BP (biological process) is represented by circles, CC (cellular component) is represented by triangles, and MF (molecular function) is represented by squares. The size of the graph represents the number of enrichments, the color represents the degree of significant difference, and the color of the *p*-value changes from green to red from large to small.

**Figure 4:** DEMs weighted gene correlation network analysis. WGCNA scale-free network distribution (a). Hierarchical clustering tree (b). Module-feature relationships validated WGCNA for correlation analysis between modules and TNM stages (d). Each row in the table in (d) corresponds to an ME, and each column corresponds to a TNM staging index. The numbers in each cell indicate the corresponding correlation and *p*-value. Cells are colored according to correlation and color legend. The strength and direction of the correlation are shown in the heatmap in the right panel (red for positive correlation and blue for negative correlation). ME : modular eigengenes.

**Figure 5:** DEGs weighted gene correlation network analysis. WGCNA scale-free network distribution (a). Hierarchical clustering tree (b). Heat map of correlation analysis between clustered modules and modules (c). Validation of WGCNA with module-feature relationship for correlation analysis between modules and TNM staging (d). Each row in the table of (d) corresponds to an ME and each column corresponds to a TNM staging indicator. The number in each cell indicates the corresponding correlation and *p*-value. Cells are colored according to the correlation and color legend. The strength and direction of the correlation are shown in the heat map in the right-hand panel (red indicates positive correlation and blue indicates negative correlation). ME: module characteristic genes.

**Figure 6:** Targeting network of LUAD miRNAs in relation to mRNAs. MiRNAs in M-phase in relation to mRNAs (a). MiRNAs in N-phase in relation to mRNAs (b). MiRNAs in Stage in relation to mRNAs (c). MiRNAs in T-phase in relation to mRNAs (d). Red is up, and blue is down.

**Figure 7:** Screening of key genes. Cytoscape analysis of DEGs in MEgrey60 module (a). Cytoscape analysis of DEGs in MElightcyan module (b). Cytoscape analysis of DEGs in MEsalmon module (c). DEGs in MEyellow module Cytoscape analysis (d).

**Figure 8:** OS analysis of 11 key genes in LUAD (based on TCGA data in GEPIA). The expression levels of (a) KIF23, (b) CDT1, (c) CDCA8, (d) CCNB2, (e) ITGB3, (f) DAPK1, (g) CDH13, (h) CDH1, (i) NCAPG, (j) KIF2C, and (k) CDC45 were highly correlated with the OS rate of LUAD patients.

## Data Availability

All data, models, and code generated or used during the study appear in the submitted article.
